RETRACTED

# The Construction of Civics in University English Courses in the New Media Environment

**DOI:** 10.1155/2022/7737504

**Published:** 2022-09-09

**Authors:** Xiaohang Ding

**Affiliations:** School of Foreign Languages, Inner Mongolia Minzu University, Inner Mongolia Autonomous Region, Tongliao 028000, China

## Abstract

The traditional education system has obvious limitations, relying on civics curriculum to cultivate and spread the national spirit. By analyzing the characteristics and goals of English courses under the new media, actively forming a large-scale ideological and political education model, and encouraging the innovation and optimization of English courses, new concepts of three-dimensional development can be proposed from the microlevel, and the coverage of ideological and political education can be expanded. Intelligent information technology can realize the coordinated development and collaborative application of English curriculum and ideological and political education. The combination of implicit education and explicit education and the combination of curriculum thinking and thinking curriculum can truly build the higher education model required by the development of the times.

## 1. Introduction

The development of curriculum thinking education has been developed for many years, but the phenomenon of silo of thinking education still exists. The integration of English language education with the Civic Education can help to build a comprehensive education system, and the relationship between the implicit and explicit education of Civic Education can be correctly handled, which can build a three-dimensional education pattern [1]. Students have more opportunities to be exposed to diversified cultures, and the integration of Civic Education can solve the phenomenon of cultural aphasia in English education, expand educational resources, realize the reshaping of values, enhance the relevance of Civic Education and English education, and build a nurturing system and nurturing mechanism with Chinese characteristics [2, 3]. New media break the limitation of time and space, realize multimodal information dissemination such as language, text, sound, and image, break the real and virtual boundaries, and its personalized features and community characteristics allow people to create personalized learning and life styles, freely join communities of interest, and form their own learning communities and life communities [4].

New media provides powerful technical support for English teaching, teachers can use communication media to change the traditional teacher-student single interaction mode, which is mainly taught by teachers, to a multidimensional interaction mode, which is mainly for students' independent learning, adopt online and offline hybrid teaching, use multimedia information to enrich classroom teaching content, and improve students' new media literacy [5]. However, while forming a team of teachers to cope with the pressure of lesson preparation, college English teachers should avoid overusing new media, issuing excessive learning tasks to students, and avoiding the entertainment of college English classes. The main features of college English course Civics under the new media perspective are: Concealment Curriculum Civics and Civics courses have both similarities and differences. While the Civic Studies curriculum promotes students to establish correct values and moral concepts through diversified means, Curriculum Civic Studies highlight the nurturing function of the diversified curriculum through indirect forms, using the professional curriculum as a carrier, and therefore has a certain concealment [6].

RETRACTED

Most of the teaching modes are carried out in an explicit way, but the curriculum thinking and politics will highlight the nurturing function in an implicit way, and the integration of thinking will also make the implicit thinking and politics education throughout the whole process of education to achieve the synergistic development of English curriculum and curriculum thinking and politics [7]. The combination of implicit education and explicit education, and the combination of curriculum thinking and thinking courses, can truly build the higher education model required by the development of the times.

## 2. Related Work

Curriculum Civics was first proposed and practiced in Shanghai universities, and it has been recognized by most universities and has become a popular topic, as in Figure 1. Many experts are engaged in the research in various professional courses, striving to comprehensively master the scientific content, grasp the theoretical basis, and systematically plan the ideological and political path of curriculum implementation, which is significant.

Since 2018, the research papers about college English and Curriculum Civics have increased significantly, as shown in Figure 2, and more and more ideological and political educators as well as college English teachers have published articles in journals, putting forward many constructive opinions on the reform of Curriculum Civics teaching of college English [11].

In today's deeply developed economic globalization, foreign languages are an important tool for young students to understand the world. The domestic research on university English courses under the perspective of curriculum thinking politics are: first, the construction of foreign language curriculum thinking politics is discussed from the macro aspect. In Reference [12], it argues that it is necessary to realize the paradigm shift from extroverted intercultural education to introspective moral education, from a one-sided focus on humanities education to both humanities and science education, and from the cultivation of cultural quality to the cultivation of discernment and communication skills, so as to contribute to the goal of comprehensive development of human education. In Reference [13], it proposed that an accurate understanding of the scientific connotation of “moral education” is the primary prerequisite for the construction of foreign language curriculum thinking and politics, and explained the specific implementation process and methods of foreign language curriculum thinking and politics from five aspects: moral, academic, technical, artistic, and benevolent. In Reference [14], it discusses the construction of foreign language “curriculum thinking politics” in terms of connotation, principles and, construction paths. Secondly, the construction of the English language course in the university is studied from the aspect of teaching materials and teaching contents. In Reference [15], it considers that the construction of teaching materials and contents is the carrier and important prerequisite for the teaching of foreign language courses, and discusses the principles, importance and strategies of the construction of teaching materials and contents. The concept and characteristics of the revision of the “New Target College English” comprehensive course are discussed meeting the needs of “establishing moral education.” In Reference [16], it proposes a discourse analysis based on the analysis of English textbooks from the perspective of thinking about politics, so as to explore the political components in nonpolitical discourse.

RETRACTED

## 3. The Construction and Evaluation of Civic Politics in University English Courses

Education is a national development plan for a hundred years. As a talent training base, universities should actively take up the responsibility of nurturing people, making it their responsibility to train socialist successors, highlighting the Party's overall leadership of the school, guiding students to develop ideals and beliefs in their formative years, and enhancing their sense of patriotism and commitment. English is a language and communication tool, using language education as a carrier to strengthen ideological education, which helps college students to develop comprehensively. As China is in a critical period of reform, the education model and education philosophy are being transformed and optimized.

The construction of university English courses will form a synergistic effect, spiral upward, and play the overall effect of “1 + 1 > 2,” and integrate the core socialist values, the spirit of thinking and discernment, national sentiment, and behavioral habits into the teaching process course in a subtle form, thus forming the design idea of university English courses' thinking and politics (as Figure 3), and achieving the construction goal of value shaping, knowledge transfer, and ability cultivation.

In the practice of college English course Civics, the traditional single instrumental evaluation (mainly examining students' English listening, reading, writing, and translating abilities) cannot reflect the Civics effect of teaching, so it is necessary to modify the course evaluation criteria and appropriately increase the proportion of process assessment, and the methods are shown in Table 1.

The textbooks are the main carriers of teaching contents. At present, the textbooks used for teaching English in domestic universities are mainly written by native English authors, which place teachers and students in foreign cultural contexts and discourse systems, and ideology is often hidden in the cultural contexts and discourse systems. In such a situation, the construction of the ideology of the curriculum requires “analysis, selection and addition” of the selected textbooks, and adherence to the principles of “student development as the center, subject attributes as the guide, and school characteristics as the basis” [17]. The principle of “student development as the center, subject attributes as the guide, and school characteristics as the basis.”

“Student development-centered” means that the teaching content should be relevant to the real social context in which students live, promote student engagement, pay attention to learning effects and feedback, and focus on Chinese students' core competencies and values, as shown in Figure 4. Therefore, the content of curriculum Civics teaching should be more based on the cultural background of Chinese English learners and reflect traditional Chinese culture and the concept of scientific development in the new era.

“Guided by the attributes of the discipline” means that the construction of curriculum thinking in university English courses needs to respect and demonstrate the characteristics of the English discipline. English as a language is itself the content, way, and goal of university English teaching. And language is the carrier of culture and consciousness, which itself has value orientation.

“Based on the characteristics of the school” means the construction of curriculum thinking and political content according to local development goals, school type, and positioning, combined with the school's school characteristics. Our university is a business undergraduate institution in Guizhou, training students mainly in economics and management, but also including engineering and art majors; so our university English course Civics teaching can increase the Civics content of business ethics, management ethics, scientific spirit, aesthetic consciousness and so on.

RETRACTED

The Civics teaching content of our university English courses includes the following modules: national policies, provincial conditions, Chinese culture, professional ethics and law, mental health, labor, and aesthetic education.  Table 2 shows the content of the English course in our university.

## 4. Case Study

This study mainly adopts the interview method to conduct structured interviews with 27 teachers who teach English courses in the researcher's school. The interview questions focused on the following three dimensions: the problems and suggestions in the construction of “Course Civics.” Among the interviewees, 78% were lecturers or above, 67% were teachers with more than 10 years of teaching experience, and 52% were communist party members, as in Table 3 and Figure 5.

### 4.1. The Current Situation of the Construction of Curriculum Thinking Politics

This section explores the respondents' awareness and implementation of the course philosophy and politics. The data show that all 27 respondents have received training related to the course thinking and politics at school level or above, and believe that all course teachers should take the responsibility of teaching students thinking and politics, and approve of the necessity of integrating thinking and politics education. 19 teachers said they would often incorporate the ideological education in the teaching of college English, and 8 teachers said they would only occasionally reflect the ideological elements consciously. As to which part of the teaching process should be integrated with political education, most of the teachers thought it should be integrated with the teaching content organically. As for the suitable elements of thinking and politics in college English teaching, the teachers expressed their views on world view, life view, political view, legal view, moral view, and excellent cultural education. Meanwhile, in the teaching methods, teachers mainly mentioned real case sharing and discussion-based teaching.

### 4.2. The Role of New Media on the Construction of Curriculum Thinking and Politics

When respondents were asked about the role of “new media + education” in the construction of English language courses, most of them said they had not considered this issue, but some of them said that the advantages of new media can expand the breadth and depth of the construction of courses. At the same time, it helps to innovate the means and forms of politics education, which can break the limitations of traditional classroom.

RETRACTED

The subjects of this study: (a) 700 first-year undergraduate students of a polytechnic university who were not majoring in English. The university has stratified the teaching of English according to the first-year students' entrance English test scores. The subjects of this study covered students of different levels and majors; (b) There were 22 university public English teachers at this university, including 8 associate professors and 14 lecturers.

An online questionnaire was distributed to non-English first-year undergraduates in our university, and 700 questionnaires were received. The questionnaire consisted of 12 multiple-choice questions. Interviews were conducted with randomly selected respondents from our university English teachers. The interviewers were in teams of two, one asking questions and one taking notes. Each interview lasted about 10 minutes and was conducted in a combination of offline and online formats. The actual number of interviewees was 22, and the content of the interviews was mainly about what teaching needs there are when integrating Civic education into university English teaching.

#### 4.2.1. About the Civic Political Element in College English Courses

*(1) Course Content*. In order to better serve students' professional characteristics, there are two main branches of college English courses in the researcher's institution: college English for arts and sports and college English for nonarts and sports, and this study mainly focuses on the course of college English for arts and sports. University English for arts and sports consists of four sub-courses: University English 1 and University English 2 are required courses, and University English 3 (English exam training) and University English 4 (Chinese cultural English course) are optional courses. In the first semester, there are 56 class hours, and the teaching contents are units 1, 2, 3, 4, 5, and 6 of the first book; in the second semester, there are 64 class hours, and the teaching contents are units 1, 3, 5, 6, and 7 of the second book and the English application ability test A level tutorials.

*(2) Civic and Political Elements*. This part analyzes the political elements and contents of New Beginnings College English Comprehensive Course, Volumes 1 and 2. Each unit of this textbook consists of three articles: Text A, Text B, and Cultural Focus, and the topics include university life, sports, culture, art, and family love. On the basis of language learning, according to the focus of each unit, members of the research team fully explored its ideological elements according to the goals of enhancing cultural confidence, cultivating patriotism, passing on the spirit of hard work, and establishing the awareness of dialectical materialism, as shown in Tables 4 and 5.

RETRACTED

#### 4.2.2. The Path of College English Curriculum Civics Construction

On the basis of establishing the goal of “thinking politics in courses” and analyzing the elements of thinking politics teaching, the researcher proposed the path of constructing thinking politics in university English courses in the context of new media, as shown in Table 6.

For example, when studying the article Unit 2 Cultural Focus: High Mountain and Flowing Stream in Book 1, the teacher combined the features of the article with “Chinese culture” and “friendship” and issued a preclass task: students worked in small groups to collect information about Two Springs Reflect the Moon, Ambush on All Sides, and the Chinese culture. Before the lesson, the teacher tapped into the two perspectives of “Chinese culture” and “friendship” and issued a preclass task: students worked in groups to collect information about Two Springs Reflect the Moon, Ambush on All Sides, High Mountain, and Flowing Stream according to the outline and streamed and uploaded their questions to the online discussion forum. In the lesson, students shared their results in small groups, and the teacher consolidated and summarized the information collected by students and answered their questions. Afterward, students were guided to retell the story through keyword prompts. After the lesson, students uploaded the audio and shared their stories of friendship on the online platform, while students assessed each other and the teacher uploaded related extension materials and wrote a reflection journal and evaluation.

#### 4.2.3. Questionnaire Data and Analysis

Among the students who participated in the questionnaire, 52.16% were male students and 47.83% were female students. The purpose of the question was to investigate whether the students agreed with the necessity of integrating Civic Education into English education in college. It was found that 83.61% of the male students thought it was necessary to integrate Civic Education; 87.16% of the female students held the same opinion, as shown in Table 7.

The main purpose of the survey on students' English proficiency was to investigate whether the level of English proficiency affects students' attitudes toward integration into Civic Education. Among the students who participated in the questionnaire survey, 48.86% had passed the English IV exam for college students. Among the 357 students who did not take the Level 4 exam, 35.47% strongly agreed and 50.56% agreed with the idea, totaling 86.03%. The survey found that the level of students' English proficiency did not significantly affect their attitudes toward the integration of Civic Education, as shown in Table 8.

RETRACTED

In this survey, 98% of the students agree that cultural communication is a two-way street, 97.72% of the students think they need to study Civic Education at the university level, and 84.72% of the students think they do not know enough about Civic Education.

Students showed individual differences in the content of interested Civic Education, with 73.71% choosing history as the cultural content of interest, 68.71% choosing art, 68% choosing literature, and 59.29% choosing folklore. This shows that most of the students are willing to learn and interested in the above four cultural aspects; about 30% of the students also chose politics and philosophy, and 6.86% of the students expressed interest in other aspects. The survey on students' self-assessment of their ability to express their thinking and political education in English shows that 46.43% of students think their ability to express their thinking and political education in English is average, 32.14% think their ability is not good, and 14% think their ability is very bad, which means that a total of 92.57% of students' ability to express their thinking and political education in English needs to be improved. The study found that 62.86% of the students' classes in our university English teaching have introduced the Civic Education, and 37.14% of the students' classes have not introduced Civic Education. The most popular ways of integrating the Civic Education are the comparison of Chinese and Western cultures, the introduction of Civic Education, the expansion of textbook content, the introduction of elective courses, and others, as shown in Table 9.

Based on the fact that most students agree with the integration of Civic Education, the next question in the questionnaire concerns students' favorite content of Civic Education integration, in the order of art, literature, history, folklore, philosophy, politics and others, as shown in Table 10.

Students generally think that the integration of Civic Education in college English education can help improve language use ability, intercultural communication ability, cultural confidence, and cultural communication ability, as shown in Table 11.

## 5. Conclusion

Citizenship education runs through the whole process of higher education and is conducive to the construction of education with Chinese characteristics. Educators must strengthen the importance and emphasis on ideological and political elements, rely on curriculum thinking and politics, and solve the current state of separation of teaching and teaching, in order to achieve the all-round development of the new era of youth. The survey found that most students are willing to learn and are interested in learning the above four cultural aspects; about 30% of the students also chose politics and philosophy, and 6.86% of the students expressed interest in other aspects. The integration and innovation of the two help to improve the traditional English and civic education pattern, through accumulation and improvement, which has brought special education into a stage of leapfrog development.

RETRACTED

## Figures and Tables

**Figure 1:** Overall trend analysis of the volume of papers published in curriculum civics.

**Figure 2:** Analysis of the overall trend of the amount of civic and political articles issued in the course of “College English.”

**Figure 3:** The goal of the construction of university English courses in thinking and politics.

**Figure 4:** Core competencies and values for students in China.

**Figure 5:** Students' scores in different sections.

**Table 1:** Evaluation methods of “College English” courses.

	Appraisal method	Assessment content	Percentage (%)
	Preclass group reading circles	Individual pre-reading, group reading circle task preparation, reading and thinking on the topic of Civics, asking questions	10

Process assessment	In-class group reading circle task sharing	Group members share their tasks in the reading circle, discuss problems, and solve them	5

	Stage tests	Unit-related English language applications such as listening, reading, writing, and translating	20

	Others	Attendance, class participation, etc	5

Summative assessment	Final exam	Knowledge of language, reading comprehension, and thinking skills learned during the semester	60

**Table 2:** Civic and political content modules of university English courses.

Module	Main content	Parenting goals
Province	Red story of Guizhou, English promotion of Guizhou landscape, etc.	Cultivate a sense of home and country, know and contribute to their hometown

Chinese culture	Excellent Chinese traditional culture	Passing on the Chinese culture and enhancing cultural confidence

Professional ethics and law	Civil code, business ethics, management ethics, science competitions, independent thinking skills, etc.	Cultivate professional character and behavioral habits of law-abiding, dedicated to work, honest and trustworthy, and fair

Mental health	Mental health knowledge, stress relief techniques, etc.	Improving psychological quality and promoting sound personality development

Labor education and aesthetic education	English social practice, Chinese aesthetic spirit, etc.	Promote the spirit of labor, enhance aesthetic quality, cultivate sentiment, and warm the soul

RETRACTED

**Table 3:** Basic information of the interviewees.

Gender	Male (7 persons)	Female (20 persons)	

Academic qualifications	Bachelor's degree (1 person)	Master's degree (23 persons)	Doctoral students (3 persons)

Title	Assistant professor (6 persons) Lecturer (10 persons)	Associate professor (10 persons)	Professor (1 person)

Communist party member	Yes (14 persons)	No (13 persons)	

**Table 4:** Civic and political elements in book 1 of the comprehensive course of university English for new beginnings.

Unit	Content	Civic elements
Unit 1	Text A: your first night at school	Never forget the original heart
	Text B: never too old to live your dream	Stick to your dreams, never give up
	Cultural focus confucius: the sage of sages	Chinese culture: Confucius

Unit 2	Text A: the opera singer	Self-identification
	Text B: play a violin with three strings	Hard work
	Cultural focus: high mountain and flowing stream	Chinese culture: Friendship, music

Unit 3	Text A: fashion forest	Dialectical thinking
	Text B: learn to live with curly hair	Self-confidence
	Cultural focus: oipao-a traditional Chinese dress	Chinese culture: clothing

Unit 4	Text A: dance with dad	Affection
	Text B: dance lessons	Affection
	Cultural focus: the dragon dance	Chinese culture: Customs

Unit 5	Text A: if the dream is big enough	Strive and never give up
	Text B: Michael Jordan's farewell letter to basketball	Strive, love
	Cultural focus: martial arts	Chinese culture: martial arts

Unit 6	Text A: techs best feature: the off switch	Dialectical thinking
	Text B: online writing	Technology, innovation
	Cultural focus: painting	Chinese culture: painting

**Table 5:** Elements of civics in book 2 of the comprehensive course of university English for new beginnings.

Unit	Content	Civic elements
Unit 1	Text A: drums in space	Thinking differently
	Text B: my father's music	Diligence
	Cultural focus be there just to make up the number	Chinese culture: idiom stories

Unit 3	Text A: dont stop the music, I want to dance	Persistence, hard work
	Text B: how I shamed the ballet world over “discrimination” against disabled ballerina	Equality
	Cultural focus: peacock dance of dai	Chinese culture: dance

Unit 5	Text A: Walt Disney and Steve Jobs connection	Innovation, stick to the original intention
	Text B: animation film frozen	Break through stereotypes
	Cultural focus: hero is back	Chinese culture: animation

Unit 6	Text A: the last runner	Hard work
	Text B: the true courage	Modesty
	Cultural focus: dragon boat racing	Chinese culture: custom

Unit 7	Text A: Vincent Van Gogh: the starry night	Persistence
	Text B: the artist of France	Western art
	Cultural focus: Chinese new year painting	Chinese culture: art

RETRACTED

**Table 6:** Paths for the construction of English language courses in the context of new media.

Before class	Online	Teachers	Refine the elements of Civics, publish preclass tasks, collect students' questions
		Student	Work in groups to complete related tasks

During class	Offline	Teachers	Language + civics teaching is complementary and organic
		Student	Discussion and sharing

After class	Online + offline	Teachers	Upload extension materials, write reflection journals, publish postlesson tasks, and evaluate
		Student	Complete related tasks, share, and evaluate

**Table 7:** It is necessary to introduce civic education in college English teaching.

*X*/*Y*	Strongly agree	Agree	Don't necessarily	Disagree	Strongly disagree	Subtotal	Average score
Male	135 (36.47%)	173 (47.14%)	50 (13.87%)	8 (1.99%)	2 (0.57%)	368	4.19
Female	141 (41.79%)	153 (45.37%)	38 (11.34%)	4 (1.19%)	1 (0.32%)	337	4.29

**Table 8:** It is necessary to introduce civic education in university English teaching.

*X*/*Y*	Strongly agree	Agree	Don't necessarily	Disagree	Strongly disagree	Subtotal	Average score
Score of 600 or above	16 (38.09%)	17 (40.48%)	7 (16.67%)	1 (2.38%)	1 (2.38%)	42	4.09
Score of 550 or above	48 (39.67%)	53 (43.80%)	18 (14.88%)	2 (1.65%)	0 (0.00%)	121	4.25
Score of 500 or above	55 (45.45%)	50 (41.32%)	14 (11.57%)	2 (1.65%)	0 (0.00%)	121	4.32
Score of 425 or above	27 (45.00%)	22 (36.67%)	8 (13.33%)	3 (5.00%)	0 (0.00%)	60	4.27
Did not take the Level 4 exam	126 (35.29%)	180 (50.42%)	46 (12.89%)	2 (0.56%)	3 (0.74%)	357	4.21

**Table 9:** Which of the following ways do you like to introduce civic education in university English teaching?

Options	Subtotal	Proportion (%)
Expansion based on textbook content	322	45.79
Introduction to the topic of Chinese culture	415	59.79
Topics on the comparison of Chinese and Western cultures	475	67.72
Introduction to English in Chinese elective course	285	40.63
Introduction to English in Chinese elective course	12	1.55

**Table 10:** Which aspects of civic education do you like to introduce in the teaching of English in college?

Options	Subtotal	Proportion (%)
Politics	178	25.32
History	472	67.37
Literature	485	69.42
Art	508	72.31
Philosophy	504	28.97
Folklore	414	59.43
Other	25	3.87

**Table 11:** Which competencies do you think will be improved by introducing civic education in college English education?

Options	Subtotal	Proportion (%)
Language use ability	547	77.87
Cultural communication ability	531	76.25
Intercultural communication ability	542	77.59
Cultural confidence	535	76.59
Other	19	2.63

RETRACTED

## Data Availability

The raw data supporting the conclusions of this article will be made available by the authors, without undue reservation.
